The article "Biofilm Formation by Pathogens Causing Ventilator-Associated Pneumonia at Intensive Care Units in a Tertiary Care Hospital: An Armor for Refuge" was published in 2021. Journal: Biomed Res Int.

# Biofilm Formation by Pathogens Causing Ventilator-Associated Pneumonia at Intensive Care Units in a Tertiary Care Hospital: An Armor for Refuge

**DOI:** 10.1155/2021/8817700

**Published:** 2021-05-28

**Authors:** Sujata Baidya, Sangita Sharma, Shyam Kumar Mishra, Hari Prasad Kattel, Keshab Parajuli, Jeevan Bahadur Sherchand

**Affiliations:** ^1^Department of Clinical Microbiology, Institute of Medicine, Tribhuvan University Teaching Hospital, Kathmandu, Nepal; ^2^School of Optometry and Vision Science, University of New South Wales, Australia

## Abstract

**Background:**

Emerging threat of drug resistance among pathogens causing ventilator-associated pneumonia (VAP) has resulted in higher hospital costs, longer hospital stays, and increased hospital mortality. Biofilms in the endotracheal tube of ventilated patients act as protective shield from host immunity. They induce chronic and recurrent infections that defy common antibiotics. This study intended to determine the biofilm produced by pathogens causing VAP and their relation with drug resistance.

**Methods:**

Bronchoalveolar lavage and deep tracheal aspirates (*n* = 70) were obtained from the patients mechanically ventilated for more than 48 hours in the intensive care units of Tribhuvan University Teaching Hospital, Kathmandu, and processed according to the protocol of the American Society for Microbiology (ASM). Antibiotic susceptibility testing was done following Clinical and Laboratory Standards Institute (CLSI) 2017 guidelines. Biofilm formation was determined using the microtiter plate method described by Christensen and modified by Stepanovoic et al.

**Results:**

Significant microbial growth was seen in 78.6% of the total samples with 52.7% monomicrobial, 45.5% polymicrobial, and 1.8% fungal infection. Among the 71 isolates obtained, bulk was gram-negative (*n* = 64, 90.1%). *Pseudomonas aeruginosa* (31.0%) was the predominant isolate followed by *Acinetobacter calcoaceticus baumannii* complex (16.9%), *Klebsiella pneumoniae* (16.9%), *Citrobacter freundii* (15.5%), *Staphylococcus aureus* (7.0%), *Escherichia coli* (5.6%), *Citrobacter koseri* (2.8%), *Enterococcus faecalis* (1.4%), *Burkholderia cepacia* complex (1.4%), and *Candida albicans* (1.4%). Of the total isolates, 56.3% were biofilm producers. Multidrug-resistant (MDR) organisms, extended-spectrum *β*-lactamase (ESBL), and metallo-*β*-lactamase (MBL) producers were preeminent among the biofilm producers. The highest producer of biofilm was *P. aeruginosa* (19.7%). Among gram-negative biofilm producers, 42.2% were MDR, 21.9% were ESBL producers, and 7.8% were MBL producers.

**Conclusion:**

Gram-negative nonfermenter bacteria account for the bulk of nosocomial pneumonia. MDR, ESBL, and MBL production was preponderant among the biofilm producers. The rampant spread of drug resistance among biofilm producers is summoning novel interventions to combat multidrug resistance.

## 1. Introduction

Nosocomial infections are those infections occurring after more than 48 hours of hospital admission [1]. These infections pose a massive challenge which has fueled up the causes of hospital morbidity and mortality. Ventilator-associated pneumonia (VAP), a form of hospital-associated pneumonia (HAP), specially refers to pneumonia occurring in patients mechanically ventilated for more than 48 hours after tracheal intubation [2]. VAP is characterized by the presence of lung infiltration (new or progressive), fever, altered white blood cell count, changes in sputum characteristics, and occurrence of a causative agent [3]. These infections account for the most complications (9–27%) associated with patients in intensive care units (ICUs) receiving mechanical ventilation [4].

The major risks of VAP include length of hospital stay, exposure to ventilator, invasive procedures, host immunity, virulence of the invading microorganisms, and cross-contamination [5]. VAP develops by direct entry of the bacteria into the lower respiratory tract which may be innate oropharyngeal flora or those in the environment drew in via aspiration, pooling, and trickling of secretions around cuff, impaired ciliary action, or biofilm inside the tube [6].

In course of expanding hospital setting, prescribing antibiotics under a crippled antibiotic stewardship is habitude. VAP itself deals with resistant pathogens, and use of broad-spectrum antibiotics for its control further aggravates the condition. In a systematic review of VAP in south-east Asian countries, the incidence of VAP ranges from 2.13 to 116 per thousand ventilator days [7]. According to the systemic meta-analysis of the incidence of adult VAP in Asian countries (2018), Nepal has VAP incidence density of 21.4 per 1000 ventilator days and period prevalence of 21.7% [8]. The incidence of VAP is higher in Nepal when compared with data of developed countries. High prevalence in Nepal was reported in various studies by Shrestha et al. (34%) [9], Mishra et al. (41.6%) [10], and Lamichhane and Mishra (24.2%) [11].

Biofilm, an assemblage of microbial cells, is irreversibly associated with a surface and enclosed in a matrix of polysaccharide material [12]. The increased resistance demonstrated by biofilm-forming organisms may be contributed by the exopolysaccharide matrix, production of exotoxin thwarting host immunity, or plasmid exchange of resistant genes [13]. Biofilm formation in the endotracheal tube of ventilated patients plays a major role in the occurrence of VAP [14]. Biofilm-producing organisms are said to be associated with nearly 50% of the nosocomial infection. They cause chronic and recurrent infections that are highly tolerant to common antibiotics [15, 16]. Bacterial cells in biofilm are about 10 to 1000 times more resistant to the antimicrobial agents in contrast to their planktonic analogues [17].

Bacteriological etiology of VAP depends on the duration of mechanical ventilation. Early onset occurs within the first 4 days of hospitalization with better prognosis while late-onset VAP occurs after 5 days or more which is mostly due to MDR organism [3]. Gram-negative bacteria (GNB) like *Acinetobacter baumannii*, *Klebsiella pneumoniae*, *Pseudomonas aeruginosa*, *Escherichia coli*, and *Enterobacter* spp. are often associated with VAP [6]. Bacteria causing early-onset VAP constitute *Streptococcus pneumoniae*, *Haemophilus influenzae*, methicillin-sensitive *Staphylococcus aureus* (MSSA), antibiotic-sensitive enteric GNB like *Escherichia coli*, *Klebsiella pneumoniae*, *Enterobacter* spp., *Proteus* spp., and *Serratia marcescens* while bacteria causing late-onset VAP include multidrug-resistant (MDR) bacteria such as methicillin-resistant *Staphylococcus aureus (*MRSA), *Acinetobacter baumannii*, *Pseudomonas aeruginosa*, and ESBL producers [18].

The incidence of VAP is commendable in previous studies in Nepal. Moreover, MDR organisms have outsmarted the treatment protocols. It is evident in various studies that biofilms play an important role in the gravity of medical-device-associated infections; however, there are no adequate studies done in Nepal in the purview of VAP to the best of our knowledge. The rationale of the study was to unravel the relation of biofilm production with antimicrobial resistance.

## 2. Materials and Methods

This was a laboratory-based cross-sectional study carried out from July 2019 to January 2020 (seven months). A total of 70 lower respiratory tract samples (bronchoalveolar lavage (BAL) and deep tracheal aspirate) were taken from patients under mechanical ventilation for more than 48 hours in the intensive care units (ICUs) of Tribhuvan University Teaching Hospital (TUTH), a 700-bed tertiary care center of Nepal.

### 2.1. Inclusion Criteria

Patients admitted and put on mechanical ventilation in ICU for >48 hours were included.

### 2.2. Exclusion Criteria

Patients with pneumonia prior to mechanical ventilation or before 48 hours of mechanical ventilation were excluded.

### 2.3. Sample Collection and Processing

Samples were collected, transported, and processed for culture and sensitivity following standard laboratory protocol of the American Society for Microbiology (ASM) [19]. Biofilm formation was detected by the microtiter plate technique as described by Christensen et al. and modified by Stepanovic et al. [20].

### 2.4. Quantitative Culture

First, one tube of 5 ml of 1x phosphate-buffered saline (PBS) was labelled as “1 : 100.” To this tube, 50 *μ*l of undiluted sample was added and vortexed for 30 to 60 seconds. 100 *μ*l of “1 : 100” dilution fluid was transferred to a plate marked “×10^3^” (each colony on this plate = 10^3^ CFU/ml). Then, another tube of 5 ml of 1x PBS was labelled “1 : 10,000.” To this tube, 50 *μ*l of “1 : 100” dilution was transferred and vortexed. Then, 100 *μ*l of the “1 : 10,000” dilution was transferred to a plate marked “×10^5^” (each colony on this plate = 10^5^ CFU/ml). The inoculum was spread over each plate evenly by using a disposable plastic rod [19].

### 2.5. Identification of the Organism

The organism isolated was identified using the protocol provided by the ASM. First, gram staining of the isolates was performed. Then, catalase and coagulase tests were done to differentiate *S. aureus* from other gram-positive isolates. Growth in bile esculin agar (BEA) and 6.5% NaCl were assessed. A sensitivity test to meropenem disks was performed to differentiate *Enterococcus faecium* (resistant) from *Enterococcus faecalis* (sensitive). A panel of biochemical tests was performed to identify different gram-negative isolates (Table 1). Oxidase tests were done to differentiate gram-negative bacteria. Resistance to the colistin group of antibiotics and cotrimoxazole was used to differentiate BCC (*Burkholderia cepacia* complex) (colistin-resistant and cotrimoxazole-sensitive) from other pseudomonads.

### 2.6. Antibiotic Susceptibility Test

The antibiotic susceptibility tests of the isolated organisms were done using Mueller Hinton Agar (MHA) by the standard disk diffusion technique of the Kirby-Bauer method as recommended by CLSI [21]. The following antibiotics with specified concentrations were used: ampicillin (10 *μ*g), ampicillin-sulbactam (10/10 *μ*g), amoxycillin-clavulanic acid (20/10 *μ*g), cefixime (5 *μ*g), ceftazidime (30 *μ*g), ceftriaxone (30 *μ*g), cefepime (30 *μ*g), cefoxitin (30 *μ*g), piperacillin (100 *μ*g), piperacillin-tazobactam (100/10 *μ*g), cotrimoxazole (1.25/23.75 *μ*g), gentamicin (10 *μ*g), amikacin (30 *μ*g), imipenem (10 *μ*g), meropenem (10 *μ*g), ciprofloxacin (5 *μ*g), levofloxacin (5 *μ*g), colistin sulfate (10 *μ*g), erythromycin (15 *μ*g), clindamycin (2 *μ*g), vancomycin (30 *μ*g), teicoplanin (30 *μ*g), doxycycline (30 *μ*g), and chloramphenicol (30 *μ*g) from HiMedia Laboratories, India.

### 2.7. Microtiter Plate Method

A 0.5 McFarland adjusted standard of the bacterial suspension was diluted 100 times in Brain Heart Infusion (BHI) broth with 1% glucose. Then, 200 *μ*l of the diluted bacterial suspension was sampled into wells of microtiter plates. The test was run in triplicates. The negative control wells were sampled with sterile BHI broth only. All other procedures were performed in the same manner as the test. The microtiter plates were incubated in static condition for 24 hours at 37°C in a normal incubator. After completion of incubation, the microtiter plate was vigorously washed by physiological saline three times to remove planktonic bacteria and nonbiofilm adhesion of bacteria. The adherent bacteria were fixed with 200 *μ*l 99% methanol then emptied after 15 minutes and left to dry. Plates were stained with a 2% Hucker crystal violet stain for 5 minutes and rinsed with tap water. After complete drying, 160 *μ*l of 33% glacial acetic acid was added to dissolve crystal violet and OD was measured at 570 nm using an automated ELISA reader. Quantification of biofilm was done from negative controls, and average OD was calculated from triplicates of each isolate [20] (Figure 1).

### 2.8. Detection of ESBL

Potential ESBL producers were determined by testing with ceftazidime (CAZ, 30 *μ*g) and cefotaxime (CTX, 30 *μ*g) disk on MHA. Those isolates with zone of inhibition (ZOI) < 18 mm for CAZ or <23 mm for CTX were confirmed by the combination disk method. Two disks: one containing CAZ (30 *μ*g) alone and the other CAZ in combination with clavulanic acid (30/10 *μ*g), were placed apart. The plate was incubated at 35 ± 2°C for 16-18 hours; an increase in zone diameter of more than 5 mm around disk containing clavulanic acid than the other disk was confirmed as positive ESBL producer [21].

### 2.9. Detection of MBL

The isolates were subjected to MBL detection when meropenem was resistant (ZOI < 25 mm). The phenotypic test for MBL production was performed by the combination disk method described by Tsakris et al. [22]. In this test, two meropenem disks (10 *μ*g) were placed on MHA. To one disk, 10 *μ*l of 0.1 M (292 *μ*g) anhydrous ethylene diamine tetra-acetic acid (EDTA) was dispensed. The plate was incubated at 37°C. After overnight incubation, an increase in zone diameter of more than 5 mm around the EDTA disk compared to the meropenem disk alone was confirmed as positive MBL production.

### 2.10. MIC

Colistin strip (E-strip from HiMedia Laboratories Pvt. Ltd., Bombay, India) was used for MIC determination. A 0.5 McFarland suspension of each isolate was prepared and lawn cultured on MHA. The colistin sulfate E-strip with antibiotic concentration from 0.016 to 256 *μ*g/ml in gradient was placed onto the inoculated plate. The plate was incubated at 37°C for 24 hours according to the manufacturer's instruction. Then, the MIC value was determined.

### 2.11. Data Analysis

All data were entered in computer and analyzed using SPSS version 20.0. Tables and charts were prepared using Microsoft Excel. The chi-square test was applied to test the significance of the relation between categorical values, and the level of significance was set at *p* < 0.1.

### 2.12. Ethical Consideration

The study was conducted after taking written approval from the Institutional Review Committee of Institute of Medicine (Ref: 424(6-11)E^2^/075/76). In addition, written consent was taken from patient's local guardian for participation in the study before enrolment.

### 2.13. Limitation of the Study

This was a laboratory-based cross-sectional study conducted in a short time period of seven months, and the outcome of the patients with VAP could not be assessed.

## 3. Results

### 3.1. Demographics and Study Setup

A total of 70 samples (7 bronchoalveolar lavage or BAL and 63 deep tracheal aspirates) from patients under mechanical ventilation were assessed. Significant growth of organisms was observed in all BAL specimens (*n* = 7), while 76.2% (*n* = 48) of the total deep tracheal aspirates yielded significant microbial growth. The median age of the study population was 50 years with a range of infants below 1 year to 85 years. Male participants were preponderant accounting for 69% (*n* = 48) while female participants summed to 31% (*n* = 22) only. The highest number of significant growth was seen in the 50 to 60 years age group and infants below 1 year of age each sharing 20% of the significant growth (Table 2).

### 3.2. Distribution of Isolates according to Growth

Among the samples received, 78.6% (*n* = 55) yielded significant growth, of which 52.7% (*n* = 29) were monomicrobial, 45.5% (*n* = 25) were polymicrobial, and 1.8% (*n* = 1) were fungal infection. A total of 71 organisms were isolated of which 90.1% (*n* = 64) were gram-negative, 8.5% (*n* = 6) were gram-positive, and 1.4% (*n* = 1) was *Candida* spp.

Among the total isolates, *Pseudomonas aeruginosa* (31.0%) was the predominantly isolated organism followed by *Acinetobacter calcoaceticus baumannii* complex (ACBC) summing to 16.9% (Table 3). *P. aeruginosa* was predominant in both early- and late-onset VAP accounting for 34.8% and 37.5% of the isolates, respectively. There was a variable level of susceptibility of isolates to different groups of antibiotics and 100% susceptibility to vancomycin, teicoplanin (gram-positive), and colistin (gram-negative). In our study, less than 50% gram-negative isolates were sensitive to carbapenem.

### 3.3. Distribution of Biofilm Production

Out of the total organisms, 56.3% (*n* = 40) were biofilm producers while 43.7% (*n* = 31) were biofilm nonproducers. Among the biofilm producers, the majority were weak producers accounting for 35.2% (*n* = 25) followed by moderate producers summing to 16.9% (*n* = 12) and only 4.2% (*n* = 3) were strong producers of biofilm (Figure 2). Among the total isolates, *P. aeruginosa* (19.7%) was the major one producing biofilm followed by ACBC (9.9%) and *K. pneumoniae* (9.9%) (Table 3). Only two organisms, namely, *P. aeruginosa* and ACBC, were strong biofilm producers with the share of 2.8% and 1.4%, respectively (4.2% altogether).

### 3.4. Biofilm Production and Drug Resistance Patterns (MDR, ESBL, and MBL)

Of the total isolates, 77.5% (*n* = 55) were MDR. Among the total gram-negative isolates, 42.2% (*n* = 27) were MDR biofilm producer, 21.9% (*n* = 14) were ESBL biofilm producer, and 7.8% (*n* = 5) were MBL biofilm producer (Figure 3). MDR organisms were preeminent in both early- and late-onset VAP. There was a high prevalence of multidrug resistance in biofilm-producing organisms. However, there was no statistically significant relation between the biofilm production and multidrug resistance, ESBL as well as MBL production. There was, nonetheless, significant association between biofilm production and resistance of *P. aeruginosa* to piperacillin/tazobactam with a *p* value of 0.070 (*p* < 0.1) (Table 4) and between biofilm formation and resistance of *Staphylococcus aureus* to gentamicin and doxycycline with a *p* value of 0.025 (*p* < 0.1) (Table 5). However, no such relation was seen in the resistance pattern of Enterobacteriaceae and ACBC (Tables 6 and 7). Among the *Staphylococcus aureus* isolated, 60% (*n* = 3) were methicillin resistant (i.e., methicillin-resistant *Staphylococcus aureus* or MRSA). There was no significant association of MRSA with biofilm production as well in our study.

## 4. Discussion

Biofilm formation by pathogens is posing a threat in infection control regardless of the ample choices of antibiotics available. While the indiscriminate use of broad-spectrum antibiotics has tapered down the choices of effective drugs to combat the so-called “superbugs,” the dreary reality is worrisome due to the spread of biofilm formation. The recent upsurge of biofilm production and drug resistance among such organisms has pulled back the era of medicine by decades as we have limited choices of antibiotics left. Early detection of biofilm formation can help modulate the treatment strategies and hence reduce mortality and morbidity. In context of Nepal, no published studies that associate biofilm formation with VAP cases are present to the best of our knowledge. Our study provides an insight to the prevalence of biofilm formation in VAP.

In this study, the highest number of growth was seen in the sample from the infant age group and the 50-60 years age group each sharing 20% of the total growth. It indicates that these groups of population are vulnerable to nosocomial infections.

This study is analogous to the study of Richards et al. which concluded that the bulk of isolates in pneumonia are gram-negative aerobic organisms among which *P. aeruginosa* was the most frequently isolated [23]. This study also correlates well with a previous study in our hospital by Mishra et al. in which *P. aeruginosa* was found to be the major pathogen causing nosocomial lower respiratory tract infection [24]. However, contrary to our findings, the study by Sah et al. in the same center reported *Klebsiella pneumoniae* and *Acinetobacter* spp. as the predominant bacteria isolated in nosocomial lower respiratory tract infections [25]. Similarly, another study by Shrestha et al. in the similar setting in neurological patients observed that *Acinetobacter* spp. (55.6%) accounted for the maximum cases of VAP [26]. These variations may be due to gradual adaptation of the microbial flora over time.

In our study, 56.3% (*n* = 40) were biofilm producers while 43.7% (*n* = 31) were biofilm nonproducers. Of the total biofilm producers, 4.2% (*n* = 3) were strong producers, and 16.9% (*n* = 12) were moderate producers while 35.2% (*n* = 25) were weak producers. These findings closely resembled the study of Gupta et al. in which 40.6% of the gram-negative isolates were biofilm producers and all of them were MDR [27]. Similarly, our study is in concord with the study of Mulla and Jethwani in which 65.4% (*n* = 34) of the isolates causing VAP were biofilm producers [28].

Our study complies well with the study of Mishra et al. in the same setting (2013) in which 46.3% of the total isolates obtained from various clinical specimens were found to be biofilm producers [29]. Meanwhile, the pattern of organisms producing biofilm reported by Mishra et al. was different from our study who elucidated *Klebsiella pneumoniae* (30%) as the major biofilm-producing gram-negative isolate [29].

It is of note that, in our study, the MDR pathogens were predominant (77.5%) among biofilm producers as well as nonproducers. Among the MDR isolates, 35.3% were biofilm nonproducers while 42.2% were biofilm producers. This accords to the conclusion stated by Cepas et al. that MDR isolates may not be greater biofilm producers than non-MDR isolates. They also reported that *P. aeruginosa* from respiratory samples were more biofilm forming than those from the other types of samples [30].

In a similar study by Dumaru et al. in another tertiary care center in Nepal, 62.7% of the isolates were biofilm producers; 26.8% and 16.7% were ESBL and MBL producers, respectively. It shows escalating drug resistance as an impending threat in our country. Likewise, the same study showed a significant association between MBL production and biofilm production while no association between ESBL production and biofilm production [31]. Our study, however, could not address such statistical relation between multidrug resistance and biofilm formation.

In our study, 77.5% (*n* = 55) of the isolated pathogens were MDR. This is in concordance with the study of Khanal et al. in a hospital in Kathmandu which showed bulk of the isolates causing respiratory infection in ICU were gram-negative isolates (92.2%) and 68.8% of them were MDR. Their study concluded that *P. aeruginosa* was the highest ESBL-producing isolate, summing up to 42.8% [5]. Our study dissents with the latter fact as in our study; ACBC (10.9%) was the highest ESBL producer while *P*. *aeruginosa* (20.3%) was the most copious MDR isolate.

In our study, gram-negative nonfermenters including *P. aeruginosa* and ACBC were predominant isolates in both early- and late-onset VAP. Contrary to our study, some studies suggest that early-onset VAP is linked to high rates of infection of oropharyngeal flora, while late-onset VAP is found mostly associated with *P. aeruginosa*, ACBC, MRSA, and MDR gram-negative bacteria [3, 32]. The occurrence of MDR nonfermenters as an eminent isolate in the early-onset VAP in our study may be due to the colonization by nonfermenters during hospitalization before shifting to ICU and acquisition of mechanical ventilation. It can also be attributed to the fact that patients under critical care are exposed to indiscriminate use of broad-spectrum antibiotics during their care or prior to the critical care which may have provoked the resistance.

In a similar study done in TUTH by Shrestha et al., the bulk of the organism associated with VAP was found to be ACBC (43.47%) which grosses the second position in our study. The antibiogram of *P. aeruginosa* in their study showed high resistance to ciprofloxacin similar to our study [9]. On the other hand, the susceptibility rate of *P. aeruginosa* to cefoperazone/sulbactam and carbapenem in their study was 82% and 91%, respectively, while our study shows the sensitivity rate has fallen to 68.2% and 45.5%, respectively. This is quite infuriating because carbapenems are the drugs of choice for ESBL producing MDR *P. aeruginosa.* This situation may be attributed to wide use of carbapenems in our ICUs due to past record of high prevalence of resistant bacteria. Similarly, 35.9% of all gram-negative isolates were ESBL producers in our study which is slightly higher than the findings of Shrestha et al. which was 32.8% [9].

In the antibiogram study of gram-positive isolates, the sensitivity rate of doxycycline and chloramphenicol was commendable accounting to 60% and 80%, respectively. These isolates had low sensitivity towards ciprofloxacin, cotrimoxazole, and erythromycin probably due to rampant empirical use of these drugs.

Our study showed statistically significant association of piperacillin/tazobactam resistance and biofilm production with *p* value of 0.070 (i.e., *p* value < 0.1) in *P. aeruginosa* and similar association with gentamicin and doxycycline resistance (*p* value of 0.025) in gram-positive isolates. But, the association of biofilm production and multidrug resistance was statistically nonsignificant. This is in accordance with the study of Cepas et al. that showed despite relationships being found between individual drug resistance, there is no relation between multidrug resistance and biofilm formation [30]. It is also supported by the studies of Shrestha et al. in uropathogens [33] and Eyoh et al. [34].

However, the antibiogram study of *P. aeruginosa* and relation with biofilm formation does not concur with the study of Neopane et al. done in another tertiary care center in Nepal which found biofilm production of *P. aeruginosa* to be strongly associated with multidrug resistance and ESBL production [35]. The same study observed the resistance of ceftazidime in biofilm-producing isolates was 57.1% which in our study was 68.2%. It can roughly point at impending threat of resistance among the biofilm producers. There are studies that show significant correlation of multiple drug resistance and biofilm formation including Bardbari et al. [36]. There are other studies conducted in tertiary care centers in Nepal as well. Nepal et al. [37] and Shrestha et al. [38] unveiled high antimicrobial resistance seen in organisms producing biofilm on inanimate surfaces. These variations could be because of isolation of different strains with different propensity of biofilm formation in different studies.

The fact that biofilm in ETT causes bad prognosis of VAP is well supported by the study of Gil-Perotin et al. which detected bacteria causing VAP in ETT biofilm and ETA despite an appropriate antibiotic therapy [14]. Organisms in biofilm can bypass the antimicrobial mechanism and the host response via exopolysaccharide layer, quorum sensing, retarded growth, sequestration of resistance genes, and many other mechanisms [15, 16]. High concentration of drugs that can control biofilm organisms cannot be obtained in the human body. This can put light on the emergence of resistance among the biofilm-producing isolates due to the consistent use of antibiotics. A strong positive correlation was reported by the study of Uppe et al. between biofilm formation and occurrence of VAP as well [39].

The pathogen causing VAP and other nosocomial infections is dynamic which may greatly vary among the hospitals, at the smallest unit of wards and even within the ICUs. There is a scarcity of local data on surveillance of infection in hospitals in context of Nepal [40]. It is unwise to administer empirical therapy without proper surveillance. Shifting to the deescalation regime is a golden tool that can diminish the emanating problem of antimicrobial resistance in critical care units. Revision of the antimicrobial resistance pattern can also help attest appropriate empirical drug choice for a particular ward and hospital.

The only drug of last regime that is left in the chest of pharmaceuticals to intervene is colistin. This has brought up a global challenge to capsize the realm of so-called “superbugs.” Being a responsible medical professional, one must intend to preserve or restore the efficacy of currently available drugs. Furthermore, coating of endotracheal tubes with antimicrobial peptides or their peptidomimetics could be an option to reduce the occurrence of VAP [41].

## 5. Conclusion

This study acquainted us about the biofilm formation and its relation with drug resistance. The data support that infants and population above 50 years are more vulnerable to nosocomial infections. Gram-negative nonfermenter bacteria constituted the bulk of isolates. Over 50% of the isolates were found to be biofilm producers. The hike in multidrug resistance, ESBL, and MBL production was also preeminent among biofilm producers. There is an increase in drug resistance reported in our study compared to similar settings. This indicates emerging drug resistance among the biofilm producers that may have grave outcomes. This study advocates further research in convenient methods of detection of biofilm in vivo as well as in vitro in the routine laboratory and to look up for alternative therapies for biofilm-associated pathogens to unburden the threat of resistant pathogens.

## Figures and Tables

**Figure 1:** Detection of biofilm formation by a microtiter plate method.

**Figure 2:** Distribution of biofilm production among isolated pathogens.

**Figure 3:** Relation between biofilm production and drug resistance of gram-negative isolates.

**Table 1:** Biochemical tests for identification of gram-negative isolates.

Organism isolated	*E. coli*	*K. pneumoniae*	*C. freundii*	*C. koseri*	*P. aeruginosa*	ACBC	BCC
TSI (slant/butt)	A/A	A/A	KorA/A	KorA/A	K/K	K/K	K/K
Gas	+	++	+	+	-	-	-
OF (glucose)	F	F	F	F	O	O	O
H_2_S	-	-	±	-	-	-	-
Motility	Motile	Nonmotile	Motile	Motile	Motile	Nonmotile	Motile
Indole	+	-	-	+	-	-	-
Citrate	-	+	+	+	+	+	+
Urease	-	+	±	±	±	±	±
Oxidase	-	-	-	-	+	-	+
Lysine decarboxylase	+	+	-	-	-	-	±
Arginine dihydrolase	±	-	±	±	+	±	-
Ornithine decarboxylase	±	-	±	+	-	-	±

Abbreviation: TSI: triple sugar iron agar; OF: oxidation-fermentation test; A: acidic (yellow); K: alkaline (red); ACBC: *Acinetobacter calcoaceticus baumannii* complex; BCC: *Burkholderia cepacia* complex; O: oxidative; F: fermentative.

**Table 2:** Age-wise distribution of growth samples.

Age group	No significant growth	Significant growth
<1 year	6 (8.5%)	14 (20.0%)
1 to 10 years	0	1 (1.4%)
10 to 20 years	0	2 (2.9%)
20 to 30 years	2 (2.9%)	5 (7.1%)
30 to 40 years	0	4 (5.7%)
40 to 50 years	3 (4.3%)	3 (4.3%)
50 to 60 years	2 (2.9%)	14 (20.0%)
60 to 70 years	0	4 (5.7%)
70 to 80 years	2 (2.9%)	6 (8.5%)
80 to 90 years	0	2 (2.9%)

**Table 3:** Biofilm production by the organisms isolated.

Organism isolated	Biofilm		Total
	Nonproducer	Producer	
*P. aeruginosa*	8 (11.3%)	14 (19.7%)	22 (31.0%)
*Acinetobacter calcoaceticus baumannii* complex	5 (7.0%)	7 (9.9%)	12 (16.9%)
*Klebsiella pneumoniae*	5 (7.0%)	7 (9.9%)	12 (16.9%)
*Citrobacter freundii*	5 (7.0%)	6 (8.5%)	11 (15.5%)
*Citrobacter koseri*	1 (1.4%)	1 (1.4%)	2 (2.8%)
*Escherichia coli*	2 (2.8%)	2 (2.8%)	4 (5.6%)
*Staphylococcus aureus*	3 (4.2%)	2 (2.8%)	5 (7.0%)
*Enterococcus faecalis*	0	1 (1.4%)	1 (1.4%)
*Burkholderia cepacia* complex	1 (1.4%)	0	1 (1.4%)
*Candida albicans*	1 (1.4%)	0	1 (1.4%)
Total	31 (43.7%)	40 (56.3%)	71 (100.0%)

**Table 4:** Relation between drug resistance and biofilm production in *Pseudomonas aeruginosa.*

Antibiotics	Biofilm				*p* value
	Producer		Nonproducer		
	Sensitive	Resistant	Sensitive	Resistant	
Gentamicin	5 (35.7%)	9 (64.3%)	4 (50.0%)	4 (50.0%)	0.512
Amikacin	5 (35.7%)	9 (64.3%)	4 (50.0%)	4 (50.0%)	0.512
Ciprofloxacin	4 (28.6%)	10 (71.4%)	1 (12.5%)	7 (87.5%)	0.387
Levofloxacin	4 (28.6%)	10 (71.4%)	2 (25%)	6 (75.0%)	0.856
Ceftazidime	4 (28.6%)	10 (71.4%)	3 (37.5%)	5 (62.5%)	0.665
Cefepime	10 (71.4%)	4 (28.6%)	4 (50.0%)	4 (50.0%)	0.315
Piperacillin	7 (53.8%)	6 (46.2%)	3 (37.5%)	5 (62.5%)	0.466
Piperacillin/tazobactam	12 (85.7%)	2 (14.3%)	4(50.0%)	4(50.0%)	0.070
Cefoperazone/sulbactam	11 (78.6%)	3 (21.4%)	4 (50.0%)	4 (50.0%)	0.166
Meropenem	8 (57.1%)	6 (42.9%)	2 (25.0%)	6 (75.0%)	0.145
Imipenem	8 (57.1%)	6 (42.9%)	2 (25.0%)	6 (75.0%)	0.145
Colistin	14 (100.0%)	0.0%	8(100.0%)	0.0%	

**Table 5:** Relation between drug resistance and biofilm production in *Staphylococcus aureus.*

Antibiotics	Biofilm				*p* value
	Producer		Nonproducer		
	Sensitive	Resistant	Sensitive	Resistant	
Ampicillin	0	2 (100.0%)	0	3 (100.0%)	
Cephalexin	1 (50.0%)	1 (50.0%)	1 (33.3%)	2 (66.7%)	0.709
Cotrimoxazole	0	2 (100.0%)	1 (33.3%)	2 (66.7%)	0.361
Gentamicin	0	2 (100.0%)	3 (100.0%)	0	0.025
Ciprofloxacin	0	2 (100.0%)	0	3 (100.0%)	
Levofloxacin	0	2 (100.0%)	0	3 (100.0%)	
Cefoxitin	1 (50.0%)	1 (50.0%)	1 (33.3%)	2 (66.7%)	0.709
Vancomycin	2 (100.0%)	0	3 (100.0%)	0	
Teicoplanin	2 (100.0%)	0	3 (100.0%)	0	
Erythromycin	0	2 (100.0%)	2 (66.7%)	1 (33.3%)	0.136
Clindamycin	0	2 (100.0%)	2 (66.7%)	1 (33.3%)	0.136
Doxycycline	0	2 (100.0%)	3 (100.0%)	0	0.025
Chloramphenicol	1 (50.0%)	1 (50.0%)	3 (100.0%)	0	0.171

**Table 6:** Relation between drug resistance and biofilm production in Enterobacteriaceae.

Antibiotics	Biofilm				*p* value
	Producer		Nonproducer		
	Sensitive	Resistant	Sensitive	Resistant	
Ampicillin	0	16 (100.0%)	0	13(100.0%)	
Cefixime	3 (18.7%)	13 (81.3%)	1 (7.7%)	12(92.3%)	0.390
Cotrimoxazole	4 (25.0%)	12 (75.0%)	2 (15.4%)	11(84.6%)	0.525
Gentamicin	7 (43.7%)	9 (56.3%)	7 (53.8%)	6(46.2%)	0.588
Levofloxacin	5 (31.2%)	11 (68.8%)	4 (30.7%)	9 (69.3%)	0.976
Amoxycillin/clavulanic acid	3 (18.7%)	13 (81.3%)	1 (7.7%)	12(92.3%)	0.390
Cefepime	6 (37.5%)	10 (62.5%)	4 (30.7%)	9 (69.3%)	0.705
Piperacillin/tazobactam	9 (56.2%)	7 (43.8%)	6 (46.2%)	7(53.8%)	0.588
Cefoperazone/sulbactam	10 (62.5%)	6 (37.5%)	6 (46.2%)	7(53.8%)	0.379
Meropenem	9 (56.2%)	7 (43.8%)	7 (53.8%)	6(46.2%)	0.897
Imipenem	10 (62.5%)	6 (37.5%)	7 (53.8%)	6(46.2%)	0.638
Colistin	16(100.0%)	0.0%	13(100.0%)	0.0%	

**Table 7:** Relation between drug resistance and biofilm production in *Acinetobacter calcoaceticus baumannii* complex.

Antibiotics	Biofilm				*p* value
	Producer		Nonproducer		
	Sensitive	Resistant	Sensitive	Resistant	
Amikacin	1 (14.3%)	6 (85.7%)	1 (20.0%)	4 (80.0%)	0.793
Levofloxacin	1 (14.3%)	6 (85.7%)	2 (40.0%)	3 (60.0%)	0.310
Ceftazidime	0	7 (100.0%)	0	5(100.0%)	
Cefepime	0	7 (100.0%)	0	5(100.0%)	
Piperacillin/tazobactam	1 (14.3%)	6 (85.7%)	2 (40.0%)	3 (60.0%)	0.310
Cefoperazone/sulbactam	2 (28.6%)	5 (71.4%)	2 (40.0%)	3 (60.0%)	0.679
Ampicillin/sulbactam	2 (28.6%)	5 (71.4%)	2 (40.0%)	3 (60.0%)	0.679
Meropenem	1 (14.3%)	6 (85.7%)	1 (20.0%)	4 (80.0%)	0.793
Imipenem	1 (14.3%)	6 (85.7%)	1 (20.0%)	4 (80.0%)	0.793
Colistin	7 (100.0%)	0	5(100.0%)	0	
Doxycycline	0	7 (100.0%)	0	5(100.0%)	

## Data Availability

The data supporting the findings of this study is available from the corresponding author upon request.
